# Comparative Evaluation of the Multilayer Perceptron Approach with Conventional ARIMA in Modeling and Prediction of COVID-19 Daily Death Cases

**DOI:** 10.1155/2022/4864920

**Published:** 2022-11-09

**Authors:** Moiz Qureshi, Muhammad Daniyal, Kassim Tawiah

**Affiliations:** ^1^Department of Statistics, Shaheed Benazir Bhutto University, Shaheed Benazirabad, Pakistan; ^2^Department of Statistics, The Islamia University of Bahawalpur, Bahawalpur, Pakistan; ^3^Department of Mathematics and Statistics, University of Energy and Natural Resources, Sunyani, Ghana; ^4^Department of Statistics and Actuarial Science, Kwame Nkrumah University of Science and Technology, Kumasi, Ghana

## Abstract

COVID-19 continues to pose a dangerous global health threat, as cases grow rapidly and deaths increase day by day. This increasing phenomenon does not only affect economic policy but also international policy around the world. In this paper, Pakistan daily death cases of COVID-19, from February 25, 2020, to March 23, 2022, have been modeled using the long-established autoregressive-integrated moving average (ARIMA) model and the machine learning multilayer perceptron (MLP) model. The most befitting model is selected based on the root mean square error (RMSE), mean square error (MSE), and mean absolute error (MAE). Values of the key performance indicator (KPI) showed that the MLP model outperformed the ARIMA model. The MLP model with 20 hidden layers, which emerged as the overall most apt model, was used to predict future daily COVID-19 deaths in Pakistan to enable policymakers and health professionals to put in place systematic measures to reduce death cases. We encourage the Government of Pakistan to intensify its vaccination campaign and encourage everyone to get vaccinated.

## 1. Introduction

From the beginning of this contagious coronavirus disease 2019 (COVID-19), it was acknowledged as a crisis that has negatively impacted almost all aspects of public and economic life. Due to the increasing infectious cases of COVID-19, there is also an increase in the death rate of patients, which creates a chaotic and mental disorder among humans across the globe. Predicting the behavior of contagious diseases is a major headache for both policymakers and health professionals [1, 2].

Jabardi et al. [3] utilized the autoregressive-integrated moving average (ARIMA) model to forecast the infection and death cases of COVID-19 in Iraq. They selected their model by implementing the root mean square error (RMSE) criteria. Shareef et al. [4] used four different models for analyzing the drift of COVID-19 cases in Pakistan and found the ARIMA model as an optimum forecasting model. Nesa et al. [5] utilized the ARIMA model for forecasting confirmed recovery and death cases of COVID-19 in Bangladesh. Banda [6] used the ARIMA model in predicting the cumulative confirmed cases of COVID-19. In their work, the appropriate model is selected based on the root mean square error (RMSE), mean square error (MSE), and mean absolute percentage error (MAPE).

Xu et al. [7] applied three machine learning models, namely, convolutional neural networks (CNNs), long short-term memory (LSTM), and CNN-LSTM to forecast new cases of COVID-19 and found that the LSTM has high accuracy in prognosticating new COVID-19 cases. Naimoli [8] compared the heterogeneous autoregressive (HAR) model and the ARIMA model in finding the positive rates of COVID-19 in Italy and concluded that the HAR model outperformed the ARIMA model. Chyon et al. [9] used the ARIMA model and machine learning propositions to predict COVID-19-affected individuals.

Machine learning approaches to time series modeling and forecasting seems to perform better with more accurate forecast values than those of the traditional time series models [7–9]. Therefore, more machine learning time series approaches ought to be explored.

### 1.1. Literature Review

Predictive and statistical models have been used constantly for modeling diseases and other pandemics. The conventional models used in time series analysis are ARIMA models proposed by Box–Jenkins for modeling and forecasting time series data.

Mohan et al. [10] put forward a hybrid ARIMA model to model and predict the daily confirmed and cumulative confirmed cases of COVID-19. The results showed that the modified ARIMA model outperformed the traditional ARIMA model in predicting the daily confirmed and cumulative confirmed cases. Argawu [11] applied the ARIMA model to prognosticate COVID-19 new cases in Algeria, Egypt, Ethiopia, Morocco, and South Africa. Rachman [12] and Zhang et al. [13] conducted a study to compare and forecast the vaccination of COVID-19 using the ARIMA and LSTM models. Chen et al. [14] employed three time series models to predict confirmed cases of COVID-19 for different provinces in Canada. They found out that the neural network outperformed the others in short-term forecasting. Ribeiro et al. [15] used ARIMA models, Cubist model, random forest (RF), ridge regression (RIDGE), support vector regression (SVR), and stacking ensemble learning in predicting one, three, and six days forward confirmed cumulative COVID-19 cases in ten Brazilian states. Warssamo and Sciences [16] developed the ARIMA model for analyzing verified recuperate and death cases in Ethiopia, while Sahai et al. [17] utilized the ARIMA model for estimating and predicting the infected cases from the top five countries with a high number of COVID-19 cases at a particular time frame, namely, the United States (US), Brazil, India, Russia, and Spain. Biswas [18] and Zeroual et al. [19] conducted a comparative study on the new daily cases of COVID-19 using five deep learning models to predict the number of recovered and new cases.

Li et al. [20] reported different ARIMA models for different countries to forecast coronavirus incidence, and their model was selected based on AIC criteria. Tan et al. [21] developed the seasonal autoregressive moving average (SARIMA) model for the analysis of the trend of the third wave of COVID-19 in Malaysia. Their model selection was based on the RMSE, mean absolute percentage error (MAE), and Bayesian information criterion (BIC). Rajab et al. [22] suggested an approach to predict the spread of COVID-19 in the United Arab Emirates (UAE), Saudi Arabia, and Kuwait by utilizing the vector autoregressive (VAR) model. Rguibi et al. [23] employed the ARIMA and LSTM models to forecast and predict the time evolution of COVID-19 in Morocco.

The epidemiological viewpoint on displaying contagious sickness spread includes the thought of a bigger number of demonstrating boundaries enumerating the spread of the infection and recuperation from the infection, extra compartments relating to mature classification, and other related decisions [24, 25]. An information-driven way to deal with displaying COVID-19 has likewise arisen, in which measurable and machine learning models are utilized for gauging cases, hospitalizations, passings, and effects of social separating [26, 27]. Considering machine learning approaches, forecasting by using artificial and wavelet neural networks with meteorological conditions has been studied by Guo et al. [28]. Guo and He [29] predicted confirmed death cases together with confirmed global COVID-19 confirmed cases utilizing artificial intelligence. Guo et al. [30] explored the changes in air quality from COVID-19 to the post-COVID-19 era in the Beijing-Tianjin-Tangshan region of China using the air quality index in machine learning, while He et al. [31] implemented artificial neural networks to predict monthly PM2.5 concentration in China's Liaocheng province.

It is clear from the above that there is an inconclusive approach to modeling COVID-19 death cases using ARIMA and machine learning techniques. In this study, we modeled daily COVID-19 death cases in Pakistan using the classical ARIMA model and the machine learning multilayer perceptron (MLP) model [32–35]. The models are compared using performance indicators (KPIs). The most appropriate model is selected to predict future cumulative COVID-19 deaths in Pakistan. Forecasting through the selected modeling technique will assist authorities in Pakistan to observe the daily death trend due to COVID-19 in Pakistan, thereby providing them with a valid tool for controlling the effects of the pandemic. This will, in the long run, help Pakistan authorities to put in place strategic prevention measures and mechanisms to curtail death cases in the country. It will also assist the authorities concerned to ascertain the intensity of the pandemic in future. Our proposed model can be compared with existing models in the literature to show predictive strength and accuracy.

The remainder of the article is organized as follows: in the upcoming section, we present the data and methods, followed by the results and discussion. In the last section, we present the conclusions of the study.

## 2. Data and Methods

### 2.1. Data

The data consist of daily confirmed COVID-19 death cases from February 25, 2020, to March 23, 2022, which are available on the official website of the Pakistan Ministry of National Health Services, Regulation and Coordination (https://covid.gov.pk). The data were collected by a joint action between the Government of Pakistan, the Pakistan Ministry of National Health Services, Regulation and Coordination, and the World Health Organization.  Table 1 shows the summary statistics of COVID-19 death cases in Pakistan.

### 2.2. Methods

#### 2.2.1. Autoregressive-Integrated Moving Average (ARIMA) Model

The ARIMA model, also known as the Box–Jenkins methodology [36], is among the best classical time series models that are used for short-term forecasting purposes. This model [ARIMA (*p*, *d*, *q*)] is a combination of three components; namely, autoregression (AR), gives us information about how the series is dependent on its past lag and denoted by a parameter *p*, the moving average (MA) part which tells us about the dependency of error terms on past lags and is denoted by *q*, and the last part is the integrated part which is used when the series is not stationary and denoted by *d*. This methodology comprises four procedures, namely, model identification, estimation of parameters, diagnostic checking, and forecasting. The series is checked by applying some tests of stationarity, and after that, the model is identified based on the correlogram of the data. It proceeds with the estimation step, and after that, the estimated models are examined based on diagnostic checking; if the candidate model fulfills the criteria, the model is utilized for forecasting. Mathematically, this model can be written as

(1) $$\begin{array}{c} \Phi_{p}\left(B\right){∆}^{d}y_{t}={ө}^{q}\left(B\right)e_{t,} \end{array}$$

if the series is nonseasonal. However, if the model is based on seasonal components, then we can write this model in terms of the backshift operator as

(2) $$\begin{array}{c} {\varphi_{P}\left(B\right)\Phi }_{p}\left(B\right){∆}^{d}{∆}_{s}^{D}y_{t}=\Theta_{Q}\left(B\right){ө}^{q}\left(B\right)e_{t}, \end{array}$$

where Φ_*p*_ stands for the autoregressive part and **ө**^*q*^ stands for the moving average part, while ∆^*d*^*y*_*t*_ denotes the difference in the series. *φ*_*P*_(*B*) is the seasonal autoregressive polynomial of order *P* and Θ_*Q*_ is the seasonal moving average polynomial of order *Q*. ∆^*d*^∆_*s*_^*D*^*y*_*t*_ is the seasonal difference.  Figure 1 shows the flowchart for this methodology.

#### 2.2.2. Multilayer Perceptron (MLP) Model

The multilayer perceptron (MLP) machine learning model [37–39] is acknowledged as one of the most flexible mathematical algorithms according to its potential applications as well as its precision in time series predicting and forecasting. The MLP model is particularly useful in approximating any type of continuous, nonlinear, differentiable, and limited function. This has made it a universal approximator. Structurally, the MLP model comprises an input layer and an output layer vis-a-vis one or more hidden layers. Artificial neurons are used to process information from one layer to another layer. Hidden layers receive the information from the input layers and then pass the information in a nonlinear function to another space, depending on the study of interest. This interconnected information then enters the output layer, resulting in the network response. The structure of the network is a feed-forward information algorithm, with connecting layers being disjoint. Mathematically, the network of the MLP model is given by the following equation:

(3) $$\begin{array}{c} y=f_{s}\left[\overset{K}{\underset{k=0}{\sum }}w_{1k}^{0}\left(f\overset{N}{\underset{n=0}{\sum }}w_{kn}^{i}u_{n}+b_{n}\right)\right]\text{,} \end{array}$$

where the network inputs *u*_*n*_ are the bias of the network *b*_*n*_, *f* is the activation function of the intermediate layers, and *f*_*s*_ is the output layer activation function. *y* is the output signal, *w*_*kn*_^*i*^ is the weight of the intermediate layer, and *w*_1*k*_^0^ is the connection of the output neurons.  Figure 2 represents the diagrammatic structure of the MLP model.

We used both models to predict the cumulative death cases in Pakistan and compared the models based on KPIs such as the mean square error (MSE), RMSE, and MAE. Mathematical expressions for KPIs are given as follows:

(4) $$\begin{array}{c} \text{MSE}=\frac{1}{T-N}\overset{T}{\underset{t=N+1}{\sum }}{\left(Y_{t}-{\hat{Y}}_{t}\right)}^{2}\text{,}\\ \text{RMSE}=\sqrt{\frac{1}{T-N}\overset{T}{\underset{t=N+1}{\sum }}{\left(Y_{t}-{\hat{Y}}_{t}\right)}^{2}}\text{,}\\ \text{MAE}=\frac{1}{T-N}\overset{T}{\underset{t=N+1}{\sum }}\left|Y_{t}-{\hat{Y}}_{t}\right|\text{,} \end{array}$$

where *Y*_1_,…, *Y*_*N*_ and *Y*,…, *Y*_*T*_ are a partition of the data. The model with the smallest KPI is selected as the most apt for the series and used for forecasting. All analyses were performed in *R*.

## 3. Results and Discussion

Figure 3 shows the visual features of the series. It can be deduced that the series is not stationary. The correlogram in Figure 4, the autocorrelation function (ACF), and the partial autocorrelation function (PACF) plot confirmed that the series is not stationary. We applied the augmented Dicky–Fuller test of stationary at a 0.05 significant level to the following hypotheses:

(5) $$\begin{array}{c} H_{o}:\text{the series is not stationary,}\\ H_{1}:\text{the series is stationary.} \end{array}$$

The *p* value of the series was found to be 0.5385, which means we fail to reject *H*_*o*_, confirming that indeed the series is not stationary. To make the series stationary, we applied difference transformation, thereby finding the order of the candidate model. This was achieved by making a correlogram of the transformed series.  Figure 5 shows the correlogram of the transformed series. From the figure, it is easy to estimate the different candidate models, and the best candidate model is selected according to KPIs. The estimated candidate models are given in Table 2.

From Table 2, we notice that the candidate model, ARIMA (6, 1, 6), is the best fit since it has the least KPIs among the other competing models. We used this ARIMA (6, 1, 6) to prognosticate future values of everyday death due to COVID-19 in Pakistan. We also present the graph of the fitted values versus the original values of the series.  Figure 6 shows the graph of the fitted versus original series, while Figure 7 shows the forecasted values given. From Figure 7, it can be observed that by using the ARIMA (6, 1, 6) model, we get the 95% and 90% confidence interval values, with the dark blue showing 95% confidence interval values and the light blue showing 90% confidence interval values. It can be noticed that the fitted values of this model efficiently follow the original series of data, which indicates that this model is efficient with a given confidence interval to forecast the daily death cases of COVID-19 in Pakistan. Our results contradict those obtained by Shareef et al. [4].

We then applied the machine learning MLP model to predict the death cases of COVID-19. To achieve this, we set the hidden layers to find the optimum estimates.  Figure 2 shows the different candidate models of the MLP.

From Table 3, we found that the MLP model with 20 hidden layers outperforms the other candidates of MLP models. It is interesting to note that as we increase the number of hidden or intermediate layers, the KPI decreases with optimum efficiency. However, increasing the hidden layer must be done with caution as the model may not remain efficient at some point after some fixed number of hidden layers.  Figure 8 shows the fitted versus the original values, while Figure 9 shows the forecasted values for the MLP with 20 hidden layers. From the figures, we can observe that the MLP model gives us multiple horizon forecasts as it indicates that the series can behave in many but limited directions. Furthermore, the residual plot indicates that the model fits to the data very efficiently and can forecast the future values efficiently. Additionally, it can also be noticed that in comparison with the ARIMA model, all MLP models outperformed the ARIMA models in terms of the KPIs. MLP with 20 hidden layers has the lowest values of MSE, RMSE, and MAE among all models considered (i.e., ARIMA and MLP models). We can state that the machine learning model, MLP with 20 hidden layers, can be utilized to forecast efficiently the future death cases of COVID-19 in Pakistan. Our MLP model performance is similar to that of Srinivasa and Santhi Thilagam [37], Deyasi et al. [38], and Chai et al. [39].

## 4. Conclusion

The COVID-19 death cases in Pakistan have been analyzed using the classical time series ARIMA model and the machine learning MLP model. Different candidate models of both models were applied and compared using different KPIs. The KPIs used, which have been frequently used in numerous classical and machine learning time series modeling, pointed to the fact that the MLP model with 20 hidden layers outperforms all other competing models for modeling and prediction purposes. It must be noted that increasing the hidden layer should be done with caution as the model may not remain efficient at some point after some fixed number of hidden layers. The MLP model was then used to forecast COVID-19 confirmed deaths in Pakistan. This will, in the long run, help authorities to put in place strategic prevention measures and mechanisms to curtail the death cases in the country. It will also assist authorities to ascertain the intensity of the pandemic in future. Although there is a strong campaign for vaccination, people should be encouraged to take vaccination seriously. It is the responsibility of the Government of Pakistan and the whole society to make the vaccination process successful.

## Figures and Tables

**Figure 1:** ARIMA model (Box–Jenkins methodology) flowchart.

**Figure 2:** Structure of a single hidden layer of the multilayer perceptron (MLP) modeling technique.

**Figure 3:** Time series plot of daily death cases of COVID-19.

**Figure 4:** ACF and PACF of daily death cases of COVID-19.

**Figure 5:** ACF and PAF after the first difference in the daily death cases of COVID-19.

**Figure 6:** Original versus fitted values using the ARIMA (6, 1, 6) model.

**Figure 7:** Forecasted values using the ARIMA (6, 1, 6) model.

**Figure 8:** Original versus fitted values using MLP with 20 hidden layers.

**Figure 9:** Forecasted values using MLP with 20 hidden layers.

**Table 1:** Descriptive statistics of Pakistan COVID-19 confirmed deaths from February 25, 2020, to March 23, 2022.

	Daily death cases
Mean	41.00
Median	32.00
Minimum	0.00
Maximum	313.00
Variance	1445.38
Lower quartile	9.00
Upper quartile	60.75

**Table 2:** Candidate models for prediction of daily death cases of COVID-19 using the ARIMA model.

ARIMA (*p*, *d*, *q*)	MSE	RMSE	MAE
ARIMA (4, 1, 5)	446.47	21.13	11.51
ARIMA (5, 1, 5)	446.05	21.12	11.50
ARIMA (6, 1, 6)	435.13	20.86	11.45

**Table 3:** Candidate models for prediction using MLP models.

MLP	MSE	RMSE	MAE
With 5 hidden layers	396.37	19.90	11.07
With 10 hidden layers	367.71	19.17	10.54
With 20 hidden layers	354.00	18.81	10.31

## Data Availability

Daily confirmed COVID-19 data from February 25, 2020 to March 23, 2022, provided by the Pakistan Ministry of National Health Services, Regulation and Government of Pakistan, were used for this study (https://covid.gov.pk).
